The article "The gender and culture effect on the CO2 emission empirical analysis" was retracted in 2024. Reasons: plagiarism; overlap with other authors' work; copyright claims; concerns about the authorship.

# The gender and culture effect on the CO_2_ emission empirical analysis

**DOI:** 10.1371/journal.pone.0296121

**Published:** 2024-02-14

**Authors:** Yanfeng Zhang, Keren Chen, Chengjie Zou

**Affiliations:** 1 Department of Digital Commerce, Zhejiang Yuying College of Vocational Technology, Hangzhou, China; 2 Seoul School of Integrated Sciences & Technologies, Seoul, Republic of Korea; 3 Institute for Economic and Social Research, Jinan University, Guangzhou, China; Jiangsu University, CHINA

## Abstract

In recent years, the world has been facing severe challenges from climate change and environmental issues, with carbon dioxide emissions being considered one of the main driving factors. Many studies have proven that activities in various industries and fields have a significant impact on carbon dioxide emissions. However, few studies have explored the impact of gender on carbon dioxide emissions. This study aims to explore the potential impact of gender diversity on carbon dioxide emissions in the boards of directors of developed and emerging market enterprises. In addition, we also analyzed how board cultural diversity affects carbon dioxide emissions. We searched two European indices provided by Morgan Stanley Capital International (MSCI) from the Bloomberg database and conducted empirical analysis. We selected the MSCI index and MSCI emerging market index from 2010 to 2019 as samples and thoroughly cleaned up the data by removing any observations containing missing information on any variables. Statistical methods such as t-test, ordinary least squares, panel data analysis, regression analysis, and robustness testing were used for statistical analysis. At the same time, differential testing was conducted on sensitive and non-sensitive sectors, and the average representation of female boards in sensitive industries was low. The research results show that the proportion of female members on a company’s board of directors is negatively correlated with carbon dioxide emissions. This discovery is consistent with the legitimacy theory advocating for gender equality and environmental sustainability, emphasizing the importance of gender diversity in reducing greenhouse gas emissions. However, agency theory suggests that diversity may lead to internal conflicts within a company, leading to agency costs and information asymmetry. The research results show a negative correlation between board cultural diversity and carbon dioxide emissions, indicating the potential challenge of board cultural diversity. This study provides important insights for decision-makers and managers, not only inspiring corporate social responsibility and environmental policy formulation, but also of great significance for academic research in the field of climate change. Our research findings help deepen our understanding of the factors that affect carbon dioxide emissions in different sectors and countries, while also expanding the research field between gender diversity, cultural diversity, and environmental sustainability. Although this study still needs to be further expanded and deepened, it provides useful insights into the relationship between board gender and cultural diversity and carbon dioxide emissions.

The article "The gender and culture effect on the CO2 emission empirical analysis" was retracted in 2024. Reasons: plagiarism; overlap with other authors' work; copyright claims; concerns about the authorship.

## 1. Introduction

In the context of global climate change and increasingly serious environmental problems, carbon dioxide emission reduction has become an important issue of common concern to the international community. As one of the main sources of global carbon emissions, enterprises’ emission reduction actions are of great significance for controlling global temperature rise. The board of directors plays an important role in the emission reduction of enterprises, and its decisions and actions directly affect the carbon emission level of enterprises. Therefore, it is of great significance to study the impact of gender diversity of corporate boards on carbon dioxide emissions and the moderating effect of cultural factors on this impact for in-depth understanding of the influencing factors of corporate carbon emissions and formulating targeted emission reduction strategies.

Recently, the focus on the environment as well as the change of climate have markedly escalated, establishing them as paramount issues of public interest [1]. Human activities, especially carbon dioxide emissions, account for 77% of total greenhouse gas emissions [2], which have made significant contributions to environmental degradation, leading to catastrophic events worldwide. In this regard, Sikandar’s [3] study explored the different impacts of trade, renewable energy, and financial development on environmental damage, and non-linear explored the differences between developed and developing countries. This study highlights the significant differences in trade, renewable energy utilization, and financial development between developed and developing countries, as well as how these factors interact with environmental destruction. Consequently, in 1997, the Kyoto Protocol was signed which secured the commitment of participating nations to significantly reduce CO_2_ emissions. In December 2015, the Paris Climate Conference was held, during which the Paris Agreement was adopted, and this agreement aims to mitigate climate change by holding global warming below 2°C and preferably at a target of 1.5°C. Hence, participating nations are urged that reducing GHG emissions by at least40% before 2030 compared to 1990 levels [4]. The United Nations has identified how to address climate change and its impacts as one of the 2030 sustainable development goals [5].

The article "The gender and culture effect on the CO2 emission empirical analysis" was retracted in 2024. Reasons: plagiarism; overlap with other authors' work; copyright claims; concerns about the authorship.

In this era of unprecedented attention to environment and climate change, Sikandar [6] demonstrates the importance and practicality of descriptive norms and moral responsibility for environmental sustainability. Expanding the Theory of Planned Behavior (TPB) provides us with a richer perspective on understanding and addressing these challenges. Naveed [7] research emphasizes that young consumers’ intention to purchase organic food is significantly influenced by their environmental awareness and attention. This is closely related to the rise of corporate social responsibility. (CSR) and the role that enterprises play in promoting sustainable development. The significant rise of Corporate Social Responsibility (CSR) has led companies to a greater awareness of the role of themselves in promoting sustainable development [8]. Consequently, due to the intensive pressure exerted by stakeholders, they are now more committed to implementing sustainable practices that enhance their environmental performance and reputation [9]. However, it is crucial to take into account that not all firms make an equal effort towards promoting sustainable development and reducing CO_2_ emissions. Prior research has identified several factors that affect companies’ level of environmental awareness. Family businesses, for instance, tend to prioritize environmental protection to safeguard their socioemotional wealth, while a company’s board of directors and ownership traits play an influential role in its contribution to environmental conservation.

Since the boards plays an essential role in driving the decision-making process and shaping the organization’s strategic direction [10], the composition of the board is critical to the company. Fan [11] is research suggests that gender differences may affect people’s ways and attitudes towards handling electronic waste, providing us with a unique perspective on how to promote sustainable behavior among different groups through different strategies and methods. In the board of directors, women place greater emphasis on social responsibility [12] and environmental protection issues [13], while they are more inclined to use new concepts and innovative solutions. Empirical research on the board’s characteristics and their impact on environmental performance suggests that gender diversity correlates positively with companies focus on environmental issues [14]. Enterprises with strong representation on female boards are more proactive in investing in environmental change innovation. This could be attributed to women’s heightened awareness of environmental issues, greater caution, and sensitivity towards the adverse impacts of the change of climate [1]. The theory of gender socialization [15] postulates that female members are more responsive to the environmental impact of company actions.

The article "The gender and culture effect on the CO2 emission empirical analysis" was retracted in 2024. Reasons: plagiarism; overlap with other authors' work; copyright claims; concerns about the authorship.

Previous researches have established the correlation between stock markets and CO_2_ emissions [16]. The expansion of capital markets has enabled companies to grow, diversify their funding sources, enhance the confidence of consumer, and finally leading to higher energy demand as well as carbon dioxide emissions. In essence, CO_2_ emissions have significant increased with economic progress [17]. Nevertheless, the stock exchange has implemented various measures to mitigate environmental degradation by encouraging eco-friendly technologies that allow for more efficient energy consumption. Additionally, the measures taken by the stock market have led to its own efficient, and making themselves a more reliable sources of financing for renewable energy projects and clean energy initiative organizations [18]. The effects of these efforts vary between developed and emerging markets due to the different of the specific implementation background of CO_2_ reduction policies; as a result, such policies are better established in developed markets than in emerging ones [18].

This paper explores the association between the diversity of gender on corporate boards and the reduction of CO_2_ emissions in developed and emerging markets. Our research aims to investigate two primary questions: (i) whether there is a correlation between female members’ representation on corporate boards and CO_2_ emissions by using developed and emerging markets as the research background? (ii) if CO_2_ emissions exhibit a correlation with gender diversity, do they also demonstrate a relationship with corporate boards cultural diversity? Further, we analyze these relationships by classifying industries according to their sensitivity to CO_2_ emissions and examine these hypotheses across different countries and industry sectors. To substantiate our hypotheses, we utilize a panel data sample encompassing developed and emerging European nations during the period 2010–2019. Our research methodology entails employing regression models.

The purpose of this study is as follows: (i) The purpose of this study is to explore how gender diversity affects carbon dioxide emissions in corporate boards, and to find out the mechanism of gender diversity on carbon dioxide emission reduction; (ii)We hope to further analyze the role of cultural diversity in corporate boards on CO2 emission reduction, in order to reveal the difference of gender diversity on CO2 emission under different cultural backgrounds; (iii)By exploring the impact of gender diversity and cultural factors on CO2 emission reduction, we hope to provide theoretical support and practical guidance for the development of more targeted carbon emission control strategies.

The article "The gender and culture effect on the CO2 emission empirical analysis" was retracted in 2024. Reasons: plagiarism; overlap with other authors' work; copyright claims; concerns about the authorship.

The results of the empirical analysis show that in terms of CO2 emissions reduction in developed and emerging markets, women have more seats on corporate boards, and this holds true across countries and sectors. These results extend previous research on the impact of gender diversity on corporate boards and confirm pre-existing speculation that women tend to be more environmentally conscious [1, 14]. At the same time, corporate board cultural diversity may further negatively affect carbon dioxide emission reduction by influencing the decision-making process and behavioral choices of corporate boards. Improving gender balance in the board of directors can enhance environmental performance to achieve effective carbon emission control.

The importance of this research can be explained from the following aspects: (i) Raise awareness of gender diversity on board decision-making: Research on the impact of gender diversity on board CO2 emissions helps us to understand the importance of gender diversity in board decision-making. (ii)Revealing the impact of boardroom cultural diversity on CO2 emissions: Studying the impact of boardroom cultural diversity on CO2 emissions will help us understand the role of cultural diversity in environmental decision-making. By analyzing how cultural diversity affects companies’ CO2 emissions, we can make better use of cultural diversity as a resource and promote the sustainable development of companies. (iii)Promoting corporate sustainability: This study focuses on how companies can achieve sustainable development by improving gender and cultural diversity and reducing CO2 emissions. This is of great practical significance for global climate change and environmental protection. At the same time, for enterprises, through research and practice, can find an effective way to improve the competitiveness of enterprises and environmental responsibility. (iv)Provide a basis for policy formulation: The research results can provide a basis for the government to formulate relevant policies. Governments can contribute to the fight against climate change by encouraging companies to increase gender and cultural diversity and promote environmentally friendly practices. (v)Expand the research field: This study combines gender diversity, board cultural diversity and corporate carbon emissions, and expands a new perspective in the field of diversity research. At the same time, it provides new ideas and methods for studying the intersection of corporate culture, organizational behavior and environmental responsibility. In summary, the importance of this study is reflected in many aspects, from enhancing the awareness of gender diversity on board decision-making, revealing the impact of board cultural diversity on carbon dioxide emissions, to promoting the sustainable development of enterprises, providing a basis for policy formulation, and expanding the research field.

The article "The gender and culture effect on the CO2 emission empirical analysis" was retracted in 2024. Reasons: plagiarism; overlap with other authors' work; copyright claims; concerns about the authorship.

This study makes significant contributions to previous research. Firstly, we examine CO_2_ emissions and corporate board diversity directly, rather than relying on information disclosure or ESG scores. While previous research has focused on corporate social responsibility as a whole, it is essential to investigate individual aspects. We identified only a limited number of empirical studies on the emissions of CO_2_ and the diversity of gender on boards; some show no relationship [19], while others linked greater female representation on boards to lower CO_2_ emissions [20]. Nonetheless, this is the first attempt at empirically analyses developed and emerging countries with similar methodologies, enabling us to identify similarities and differences. Secondly, we provide evidence on cultural diversity on corporate boards, which researchers have not studied extensively in relation to CO_2_ emissions. While past study found no correlation between cultural diversity and CO_2_ emissions [19], an international study revealed a negative connection [21]. Thirdly, our study differentiates between sensitive sectors and insensitive sectors to CO_2_ emissions. Fourthly, we perform sector-by-sector analyses. Finally, this study first attempt at conduct country-by-country analyses.

## 2. Literature review and hypotheses

In the company, the board of directors determines a strategies, policies, and objectives, making their characteristics influential not only in organizational performance but also in its social image establishment [22].

As a crucial dimension of corporate governance mechanisms, gender diversity is widely acknowledged recently [23], and this has drawn attention from policymakers, business leaders, media, and scholars worldwide [24]. Board structure and gender diversity have a significant impact on a company’s environmental performance. As the highest decision-making body of the company, the structure of the board of directors can affect the strategic direction and decision-making process of the company [10, 25]. Several studies have shown that gender diversity on boards can lead to a reputation for superior environmental performance [26], through better strategic competence and competitiveness on environmental issues [27, 28] and Environmental Disclosure [29, 30]. Companies with more gender diversity on the board have higher environmental performance [31], greater use of renewable energy sources, and fewer prosecutions for environmental infringement. Altunbas et al. [32] found that companies with more female managers reduced carbon emissions. This may be because men are closer to realizing and gaining economic benefits, while women are closer to pursuing social values. It has also been suggested that women are more compassionate and, therefore, more involved in matters of strategic importance, for example, the concerns of stakeholders [33], including environmental and social issues [34].

The article "The gender and culture effect on the CO2 emission empirical analysis" was retracted in 2024. Reasons: plagiarism; overlap with other authors' work; copyright claims; concerns about the authorship.

At the same time, the impact of female directors on corporate environmental performance is multifaceted. Several studies have provided a global view on how female directors affect corporate environmental performance, and Galbreath’s [35] study shows that female directors can improve corporate environmental performance by pushing companies to implement more environmental protection measures. Research by Gull et al. [36] suggests that female directors can reduce a company’s environmental pollution by pushing companies to implement more waste management practices. Research by Liao et al. [37] found that female directors can improve a company’s environmental performance by pushing the company to implement more corporate social responsibility measures. However, there is little empirical research on CO2 emissions and gender diversity in the boardroom. Haque [38] found no relationship from a sample of UK companies. But a study of samples of European companies by number and Velte [20] and GarciaMartin and Herrero [39] found that an increase in the number of women on corporate boards was associated with lower CO2 emissions. This suggests that boardroom gender diversity has a positive impact on a company’s environmental performance, but more empirical research is needed to confirm it.

Globalization has resulted in corporations becoming more culturally diverse [40], which entails incorporating various perspectives, values, customs, religions, educational qualifications, information processing, and management approaches [41]. The diversity of the board of directors is defined as the heterogeneity of cultural background, race, gender skills, experience, and preferences [42]. Cultural diversity enables boards to better understand the needs and expectations of local stakeholders in different communities [43]. However, cultural diversity can lead to a decrease in the efficiency of board operations, thereby hindering the communication of various ideas and perspectives. Therefore, it is crucial to investigate the influence of the diversity of cultural on boards. While the diversity of gender on boards and its influence on company operations have been widely researched, little research has explored other variables in the board of directors, notably the diversity of cultural, particularly in developing nations [23], that influence management decisions [44].

The article "The gender and culture effect on the CO2 emission empirical analysis" was retracted in 2024. Reasons: plagiarism; overlap with other authors' work; copyright claims; concerns about the authorship.

The literature presents conflicting views regarding the impact of the diversity of cultural on boards [45]. Firstly, On the one hand, agency theory supports the view that having a large and diverse board is likely to result in issues reaching consensuses because of less effective message delivery [46]. Furthermore, the diversity of cultural may create intra-company conflicts which may lead to agency costs and asymmetry in information [47]. Conversely, resource dependency theory proposes that boards with larger scale and more diverse provide access to a wider range of useful resources via the members’ talents and connections, while also increasing their societal legitimacy. Furthermore, culturally diverse companies are believed to have more comprehensive and higher quality data. Thus, the variety of perceptions stemming from the diversity of cultural allows a more diverse board to comprehend and satisfy a broader group of stakeholders, leading to a company with an open vision [48].

There is relatively little research on the relationship between board cultural diversity and carbon dioxide emissions. Khaoula Aliani et al. [49] demonstrated that the two dimensions of board diversity (cultural and skill diversity) make a positive and significant contribution to the outstanding environmental performance of the best citizen company, leading to high CO2 emissions scores. Faizul Haque [50] examined the impact of board characteristics and sustainable compensation on carbon reduction measures and greenhouse gas (GHG) emission policies of enterprises. Board independence and gender diversity were positively correlated with carbon reduction measures. In addition, compensation policies based on environmental and social governance are positively correlated with carbon reduction measures. Christian Kreuzer et al. [51] investigated whether board characteristics (such as size, skills, independence, multiple affiliations, gender diversity, corporate social responsibility (CSR) efforts, and cultural variables) affect a company’s carbon emissions. Identifying boards with more proficient skills or a higher proportion of female members can reduce greenhouse gas emissions.

The article "The gender and culture effect on the CO2 emission empirical analysis" was retracted in 2024. Reasons: plagiarism; overlap with other authors' work; copyright claims; concerns about the authorship.

## 3. Theoretical assumption

In the context of global climate change and sustainable development, it is important to study how gender diversity in corporate boards affects CO2 emissions. As a result, various theories have emerged to explain how gender-centric business practices affect different aspects of company behavior. Among these theories, resource dependence, socialization, social role, stakeholder agency theory, stakeholder theory, agency and legitimacy are noteworthy.

Although existing studies have shown that gender diversity of corporate boards can affect corporate carbon emission behavior, there are still some shortcomings in existing studies. First of all, most studies focus on western developed market countries, and there is relatively little investigation on emerging market countries. Secondly, the research method is relatively simple, lack of comparative analysis and empirical test, resulting in the reliability and universality of the conclusion is questioned. Therefore, this paper aims to fill this research gap and provide a more comprehensive and in-depth understanding of the impact of gender diversity on corporate CO2 emissions.

Gender socialization theory posits that the early life experiences of females foster a heightened awareness of issues confronting others, rendering them more attentive to ethical and environmental considerations than men. In a business, male and female directors may be influenced by different factors when making decisions. For example, female directors may be more concerned about environmental protection and social responsibility, while male directors may be more concerned about the economic benefits of the company. Therefore, gender diversity can promote companies to take more factors into account when making decisions, including environmental protection and social responsibility. Women have received education to care for others, which makes them more sensitive to environmental and social challenges [52]. As such, men and women often exhibit divergent attitudes toward ethical and competitive decision-making [24]. Liu [53] affirms this contention, maintaining that firms with female members in their decision-making department are less likely to engage in fraudulent, unethical, or tax-evasive activities. Multiple surveys have underscored women’s greater concern over the risks posed by climate change [54]. Ultimately, due to their unique perceptiveness, women tend to bear greater responsibility for environmental issues and eschew illegal or immoral actions like environmental pollution [14]. At present, the prevailing view on the impact of gender diversity on corporate board CO2 emissions is that the higher the proportion of women on corporate boards, the lower the company’s carbon emissions. This view is mainly based on the advantages of women in environmental awareness and sustainable development, and the ability of women in the board to provide a more diverse perspective on the environmental decision-making of companies. However, this view does not take into account social and cultural differences in different countries and regions, industry characteristics, and corporate governance structures. Therefore, this paper will verify and supplement this mainstream view through a comparative analysis of corporate cases in developed and emerging market countries.

The article "The gender and culture effect on the CO2 emission empirical analysis" was retracted in 2024. Reasons: plagiarism; overlap with other authors' work; copyright claims; concerns about the authorship.

Social role theory posits that societal expectations and cultural norms shape gender differences rather than innate traits. Women’s unique caregiving commitments to children and households contribute to behavioral distinctions between genders, stemming from learning experiences rather than biological determinants. Gender-based beliefs and expectations influence people’s behavior, leading to varying management styles based on sex. Notably, women exhibit greater sensitivity and empathy toward stakeholder problems, including environmental concerns [37]. Thus, firms led by women in top monitoring positions prioritize stakeholder interests [24]. Both gender socialization theory and social role theory reveal how gender diversity affects organizational behavior and decision-making. For example, transformational leadership can enhance employee motivation and organizational citizenship behavior by encouraging and supporting employees, which helps shape a more inclusive and diverse organizational culture. Sikandar Ali [6] found that transformational leadership can also influence organizational performance and social responsibility by improving employee performance and organizational citizenship behavior. This leadership style helps drive positive organizational change, including gender diversity.

Agency theory emerged from the difference between the right of ownership and the right of control, resulting in managers acting in their self-interest and harming shareholders. According to agency theory, corporate executives’ decisions may be influenced by their own interests and personal preferences. Introducing gender-diverse members to the board can increase transparency and fairness in decision-making and reduce agency costs. Therefore, we expect that gender diversity will help reduce agency costs, which in turn will reduce the carbon emissions of businesses. Managers who wish to build an environmentally friendly atmosphere have to bear the costs incurred, which displeases shareholders and reduces their profits. One way to mitigate agency costs is through greater transparency and accountability, reducing information asymmetry. Accordingly, women’s increased presence on corporate boards of directors enhances audit performance, reducing environmentally harmful practices. We get an awareness that gender diversity leads to increased independence of corporate boards, which leads to increased commitment to environmental practices and their dissemination. Corporate boards with more female members are more likely to disclose company information, as evidence suggests.

The article "The gender and culture effect on the CO2 emission empirical analysis" was retracted in 2024. Reasons: plagiarism; overlap with other authors' work; copyright claims; concerns about the authorship.

The stakeholder theory states that involved stakeholders and other relevant parties have a vested interest in whether financial outcomes nor non-financial outcomes, which includes environmental outcomes. Enterprises should attach importance to the attention of multiple stakeholders, especially environmental innovation, which has increased the pressure of various stakeholders on the enterprise. A board with a higher degree of diversification is more likely to understand the company’s environment [55], grasp the concerns of a wider range of stakeholders, and recognize its own interests [56]. The theory posits that companies operate within society and bear responsibility for mitigating any environmental damage they have caused through their actions. Research demonstrates that women exhibit stronger moral convictions regarding corporate social responsibility, particularly concerning environmental issues, leading to companies’ increased willingness to satisfy stakeholder demands [31]. Stakeholder theory holds that companies should not only pay attention to the interests of shareholders, but also to the interests of other stakeholders, such as employees, customers, suppliers, governments and communities. As the decision-making body of the enterprise, the board of directors needs to weigh the needs and interests of different stakeholders. According to stakeholder theory, gender diversity can bring a more holistic vision to the company, allowing the board to better balance the interests of all parties when considering carbon emissions. Therefore, we expect that gender diversity will help companies adopt more responsible carbon emission strategies. Thus, the presence of female members on boards correlates with higher levels of ethical behavior and adoption of social responsibility practices, indicating a higher degree of stakeholder orientation [57].

On the basis of the above two theories, it can be deduced that the board serves not only act as the principal of the management but also play the role of the stakeholders’ agent [14], which is known as the stakeholder agency theory. Gender-diverse boards is known as an effective measure to improve information transfer between shareholders as vested interests and management as agents. The measure facilitates conflict reduction between shareholders and management, at the same time helps to enhance corporate image and reputation [31]. Moreover, studies have demonstrated that boards with a higher proportion of female members exhibit greater independence, supporting the stakeholder agency theory [31]. However, Prado-Lorenzo and Garcia-Sanchez [58] discovered that the proportion of female members on boards did not affect the disclosure of information on GHG emissions from company operations.

The article "The gender and culture effect on the CO2 emission empirical analysis" was retracted in 2024. Reasons: plagiarism; overlap with other authors' work; copyright claims; concerns about the authorship.

The adoption of social media and gender diversity in the board of directors are two important issues in current business practice. Both issues are related to the company’s strategic decision-making, organizational performance, and social responsibility. Sikandar’s research shows that through the adoption of social media, SMEs can improve their marketing strategies and enhance interaction with consumers and other stakeholders. Both agency theory and stakeholder theory highlight the importance of gender diversity in board governance and corporate social responsibility practices. As Sikandar’s research shows, the adoption of social media is also a key factor affecting the performance of small and medium-sized enterprises (SMEs) [59]. These studies indicate that social media, as a powerful tool, can promote interaction and communication between companies and stakeholders, thereby improving transparency and accountability in enterprises. Combining agency theory and stakeholder theory, we can see how social media plays a mediating role between board gender diversity and corporate performance [60]. By adopting social media strategies, boards of directors with gender diversity can better communicate with stakeholders, reduce information asymmetry, reduce agency costs, and thereby improve corporate social responsibility and environmental performance. On the other hand, a board of directors with gender diversity can bring a broader perspective and more comprehensive decision-making, which helps companies make better decisions in terms of ethics and social responsibility [24]. Sikandar’s study takes into account the impact of technological, organizational, and environmental factors on social media adoption, indicating that these factors are closely related to corporate governance and gender diversity. From this, we can further explore how to promote organizational environmental sustainability strategies and practices through gender diversity in the board of directors and effective use of social media. While all of the above theories point to a relationship between environmental measures and board diversity, such as reducing CO_2_ emissions, legitimacy theory and Stakeholder theory offer the strongest reflection of this association.

The article "The gender and culture effect on the CO2 emission empirical analysis" was retracted in 2024. Reasons: plagiarism; overlap with other authors' work; copyright claims; concerns about the authorship.

Legitimacy theory contends that the quantity of CO2 emissions reflects a company’s ethical legitimacy. While reducing emissions is expensive for firms, doing so can enhance social acceptability, potentially yielding advantages such as increased sales and improved credit access. In conclusion, lowering emissions can boost financial performance, while female board members can augment corporate legitimacy by two means. For one, women’s unique psychological traits render them more attuned to stakeholder concerns, fostering better CSR outcomes [61]. Alternatively, by increasing company resources, female directors can enhance the firm’s financial capabilities to mitigate emissions and fulfil stakeholder demands. Legitimacy varies by context; what is acceptable in one industry may not be so in others [62]. Furthermore, cultural differences can impact varying stakeholder perspectives, and standards of legitimacy may diverge across countries. Hence, evaluating whether our hypotheses retain validity in varied industries and regions is crucial [63, 64].

Stakeholder theory can provide theoretical support for this research, because the board of directors will consider the needs and expectations of stakeholders when making decisions. In this study, gender diversity as one of the stakeholders may influence board decisions on CO2 emissions. Gender diversity can bring different perspectives, experiences and expertise, which may enable boards to consider CO2 emissions more holistically. In addition, stakeholder theory also emphasizes corporate responsibility to society and the environment, which makes the impact of gender diversity in the board even more important.

Legitimacy theory and stakeholder theory are two commonly used theoretical models in the field of corporate social responsibility, which have wide applicability and can be used to analyze corporate environmental responsibility and social responsibility. Therefore, these two theoretical models are very suitable for analyzing the impact of gender diversity and board cultural diversity on corporate CO2 emissions.

Specifically, legitimacy theory emphasizes that companies must adhere to social norms and values in order to gain social acceptance and support, otherwise companies may face reputational and economic risks. In the field of environmental responsibility, the environmental legitimacy of enterprises is particularly important. Therefore, the legitimacy theory can be used to analyze whether the environmental protection behavior of enterprises is based on the obligation to comply with social norms or to obtain social recognition. Stakeholder theory emphasizes that enterprises should realize sustainable development by paying attention to the needs of stakeholders. The stakeholders facing enterprises include shareholders, employees, customers, society and other aspects. In the field of environmental responsibility, enterprises also need to consider the impact of environmental protection on employees, customers and other stakeholders, as well as the contribution of corporate environmental protection behavior to the overall society. Stakeholder theory can help us better understand whether the environmental behavior and strategy of enterprises should be based on the comparative advantages of business and environmental protection or to meet the expectations of stakeholders.

The article "The gender and culture effect on the CO2 emission empirical analysis" was retracted in 2024. Reasons: plagiarism; overlap with other authors' work; copyright claims; concerns about the authorship.

In terms of adding empirical variables, we can select the appropriate variables according to the empirical research of the previous literature and the actual situation. For example, when analyzing the impact of gender diversity on corporate CO2 emissions, variables such as the proportion of women on the board and the proportion of women on the board can be added. When analyzing the impact of cultural diversity of the board of directors on corporate CO2 emissions, variables such as the proportion of directors with different cultural backgrounds and the proportion of members with different cultural backgrounds in the board of directors can be considered. The selection of these variables needs to take into account data accessibility and the explanatory power of the variables to improve the validity and reliability of the study.

From the above evidence, it is hypothesized that increasing the percentage of female members on board will lead to the reduction of CO_2_ emissions in developed as well as emerging economies. Consequently, our research posits the hypothesis as following:

**Hypothesis 1**. A negative correlation exists between the percentage of women on the board of directors and CO_2_ emissions.

Studies on group dynamics have indicated that as groups become more homogeneous, communication obstacles tend to decrease. However, this may also result in conformity to group thinking, leading to less stringent monitoring standards. This ongoing debate includes the opinions of Zaid et al. [23], who contended that the diversity of cultural on boards results in superior decisions regarding the topics of social and environmental, thereby promoting sustainable business development. Conversely, Miller and Triana [65] believe that boards with culturally homogeneous members may undermine decision-making quality by weakening constructive debates. Liao et al. [30] specially pointed out that climate-related initiatives entail a high level of complexity in their execution because they involve multiple stakeholders.

The article "The gender and culture effect on the CO2 emission empirical analysis" was retracted in 2024. Reasons: plagiarism; overlap with other authors' work; copyright claims; concerns about the authorship.

Recent empirical studies have mirrored this inconsistency in theories. For instance, Haque [50] noted that no correlation was found between the various attributes of the board of directors, while Varrone et al. [41] held a different opinion, arguing that greater diversity of board leads to superior sustainability performance. The diversity of board is often regarded as a two-pronged phenomenon, with both benefits and drawbacks. Ultimately, the relative weights of the positive and negative aspects determine the overall outcome. To further clarify this paradox, the hypothesis we propose is as follow:

**Hypothesis 2**. A positive correlation exists between board cultural diversity and CO_2_ emissions.

## 4. Dataset and methodology

### 4.1. The dataset

We conducted an empirical analysis using two European indices provided by Morgan Stanley Capital International (MSCI) which is retrieved from the Bloomberg database: the first one is the MSCI Europe index, composed of medium and large firms from 15 developed European countries, namely the Austria, Belgium, Denmark, Finland, France, Germany, Ireland, Italy, the Netherlands, Norway, Portugal, Spain, Sweden, Switzerland, and the United Kingdom. The second one is the MSCI Emerging Market (MSCI EM) Europe index, which is composed of companies from 6 emerging markets in Europe, namely the Czech Republic, Greece, Hungary, Poland, Russia, and Turkey. Thus, we conducted two separate analyses to determine if firms operating in developed countries react similarly to those in emerging countries regarding the research hypotheses. The detailed data was shown in S1 File. We conducted a sectoral analysis by differentiating between industries that are highly vulnerable or not vulnerable to CO_2_ emissions.

Our sample was taken from the MSCI index and the MSCI EM index from 2010 to 2019. The former is composed of 6,233 observations and the latter is composed of 404 observations. We conducted a thorough data cleaning process by removing any observations that contained missing information for any of the variables. This approach was adopted to enhance the validity and reliability of our findings.

Table 1 presents the mean values. As is shown by the table, the four sectors, namely Energy, basic materials, utilities, and consumer non-cyclicalare the sectors with the highest levels of CO2 emissions, while technology has the lowest level. Regarding gender diversity on corporate boards, technology, consumer cyclicals, and healthcare have the highest representation of women, while the other three sectors, namely energy, utilities, and telecommunications services have lower representation. Thus, we found that there is a negative correlation between the board’s composition of female member and the level of CO_2_ emissions. Conversely, for cultural diversity, the consumer non-cyclical as well as the utilities sectors, followed by healthcare, have the highest levels of pollution and cultural diversity.

The article "The gender and culture effect on the CO2 emission empirical analysis" was retracted in 2024. Reasons: plagiarism; overlap with other authors' work; copyright claims; concerns about the authorship.

**Table 1:** Sample description.

	Percent	CO_2_ Mean (+)	BGD Mean (†)	BCD Mean (*)
1. Basic Materials	9.615	10.365	24.195	44.125
2. Consumer Cyclicals	13.613	14.196	28.220	39.326
3. Consumer Non-Cyclicals	6.419	13.499	25.946	44.221
4. Energy	5.006	11.246	22.948	37.195
5. Financials	18.649	12.859	22.635	38.225
6. Healthcare	6.825	11.364	27.163	48.416
7. Industrials	16.329	10.226	22.956	43.645
8. Technology	6.042	10.995	28.263	46.289
9. Telecommunications Services	5.965	12.036	20.416	43.485
10. Utilities	4.023	13.416	28.529	45.241

(^+^) Mean of the logarithm of total CO_2_ and CO_2_ equivalent emission in tones.

(^†^) Mean of the percentage of women on board of directors.

(*) Mean of the percentage of members on board of directors with a cultural background different from those of the company’s headquarters.

### 4.2. Variables description

Table 2 shows the specifics of each variable, along with their corresponding abbreviations. Our dependent variable is the combined amount of CO_2_ and CO_2_ equivalent emissions in tons (CO_2_), with the natural logarithm applied to the regression coefficients’ scale. To our knowledge, no prior research has performed a comparative analysis between developed and emerging European countries.

**Table 2:** Description of variables.

Abbreviation	Variables	Definition
CO_2_	Ln CO_2_ Emission	Logarithm of total CO_2_ and CO_2_ equivalent emission in tones
BGD	Board Gender Diversity	Percentage of board members who are women
BCD	Board Cultural Diversity	Percentage of board members with acultural background different from
MTB	Market to Book	The market value divided by the book value
PER	Price Earnings Ratio	The company’s stock price divided by the earnings per share (daily time series ratio)
ROA	Return on Assets	Profit to total assets, percent
REV	Ln Revenue	Logarithm of revenue
IND	Indebtedness	Total debt to total equity, percent
PEM	Policy Emissions	Dummy variable, 1 if the company has a policy to improve emission reduction and 0, otherwise
TEM	Target Emissions	Dummy variable, 1 if the company has set targets for emission reduction and 0, otherwise
EEI	Environmental Expenditures Investments	Dummy variable, 1 if the company reports on its environmental expenditures investments to minimize future risks or increase opportunities and 0, otherwise.
PEE	Policy Energy Efficiency	Dummy variable, 1 if the company has a policy to improve its energy efficiency and 0, otherwise
BIR	Biodiversity Impact Reduction	Dummy variable, 1 if the company reports on its impact on biodiversity or activities to reduce its impact on the native ecosystems and species, as well as the biodiversity of protected and sensitive areas
IBM	Independent Board Members	Percentage of independent board members
PBD	Policy Board Diversity	Dummy variable, 1 if the company has a gender diversity policy on the board of directors and 0, otherwise
DCS	Day-care Services	Dummy variable, 1 if the company provides, day-care services and 0,otherwise
HRP	Human Rights Policy	Dummy variable, 1 if the company has a policy to ensure the respect of human rights and 0, otherwise
EGD	Executive Members Gender Diversity	Percentage of female executive
BSS	Board Specific Skills	Percentage of board members who have either an industry specific background or a strong financial background
EME	Developed/Emerging	Dummy variable, 1 if the company’s headquarters is located in an emerging country and 0, otherwise
SES	Sensitive Sector	Dummy variable, 1 if the company belong to a CO_2_ emission sensitive sector (basic materials, consumer noncyclical, energy and utilities) and 0, otherwise

Our primary independent variable and focus of analysis is the proportion of female member serving on boards, which serves as an indicator of gender diversity within monitoring roles. Prior research has established a positive correlation between the proportion of female member on boards and a higher degree of execution and disclosure of corporate social responsibility initiatives generally [1], as well as sustainable business practices specifically [20]. Nevertheless, the direct correlation between the representation of female member on boards and CO_2_ emissions, a major concern for the global community, has received limited attention in previous studies. Most of these studies have focused on the influence of women’s representation on corporate disclosure regarding greenhouse gas emissions and through empirical analysis found there is a positive association between them [66]. In contrast, there are limited number of previous studies have specifically examined the connection between women’s increased participation on boards and the level of CO_2_ emissions. These studies have reported either no correlation [50] or an inverse relationship [20].

The article "The gender and culture effect on the CO2 emission empirical analysis" was retracted in 2024. Reasons: plagiarism; overlap with other authors' work; copyright claims; concerns about the authorship.

We also examine the influence of the diversity of cultural on the composition of corporate boards as an independent variable in relation to CO_2_ emissions. This variable has only been previously analyzed in terms of its correlation with CO_2_ disclosure [70], which reported a positive association. Specifically, previous research has solely examined this variable’s connection to CO_2_ disclosure [70], finding a positive correlation between the two.

We utilized three different sets of control variables: the first one is financial market, the second one is financial accounting, and the third is environmental policy variables. The variables of financial market, which reflect investors’ long-term outlook for their firm, were analyzed. Specifically, we examined the ratios of market-to-book (MTB) and price-earnings (PER), as is typical in existing research [14, 52]. Although it may appear reasonable for the market to favor lower CO_2_ emissions, resulting in a negative correlation with the dependent variable, empirical data yield mixed results. While some studies have identified a positive correlation [67], others have found a negative relationship [58]. In addition, a significant number of studies indicated that the possible outcomes of such interactions vary with the model employed [20].

The variables of accounting reflect the current status of a corporate based on previous management decisions and events. Specifically, we utilized three accounting variables: the first one is return on assets (ROA), the second one is logarithmic revenues as an indicator of company size (REV), and the third one is debt ratio as a reflection of financial status (INDEB), following previous studies [31, 68]. Previous research has reported varying results for the correlation between these factors and CO_2_ emissions, showing differences in both direction and significance.

In their study, Valls Martínez et al. [69] utilized four dummy variables to measure a firm’s participation in corporate social responsibility initiatives: the first one is energy efficiency policy implementation, the second one is reporting on crisis management systems, the third one is receiving awards for social, environmental activities, ethical, or community, and the last one is having a CSR committee. Based on previous approach, we employ five different dummy variables to assess the environmental engagement of a company. Accordingly, we assessed whether the company had implemented measures to reduce emission (PEM), established targets for emission reduction (TEM), disclosed information on environmental expenditure as a means of minimizing potential risks or enhancing opportunities (EEI), implemented policies to enhance energy efficiency (PEE), and reported on the impact of its activities on biodiversity, including efforts to mitigate any negative consequences on native ecosystems, species, and protected or vulnerable areas (BIR). We anticipate a positive correlation between each of these variables and CO_2_ emissions.

The article "The gender and culture effect on the CO2 emission empirical analysis" was retracted in 2024. Reasons: plagiarism; overlap with other authors' work; copyright claims; concerns about the authorship.

Consistent with prior research, and recognizing the existence of targeted legal and ethical frameworks aimed at reducing the ecological impact of highly-polluting industries, we incorporated dummy variables to identify whether a company operates within a CO_2_ emission-sensitive industry [70]. We classified basic materials, consumer non-cyclical, energy, and utilities sectors as those characterized by particular sensitivity to CO_2_ emissions.

Lastly, in line with our research objective, we incorporated a dummy variable to discern whether a company operates within a developed or emerging country, with the intent of examining potential links between location and CO_2_ emissions.

Prior research has tackled the issue of reverse causality between corporate social responsibility (CSR) performance and the diversity of gender on boards by employing instrumental variables to calculate the proportion of female member on boards [52]. Given that decreasing CO_2_ emissions constitutes a crucial aspect of CSR, we can utilize instrumental variables to estimate the presence of female members on boards, thus illustrating a parallel relationship between the two phenomena [20]. Quota regulations have been implemented in most European countries [14], which is probably result in a higher number of female being appointed to independent director positions, we utilized the percentage of independent board members (IBM) as an instrumental variable [14]. Firms that prioritize gender diversity within executive roles are expected to be more inclined to appoint female board members, making executive member gender diversity (EGD) a relevant instrumental variable in our examination [20]. Additionally, we include other instrumental variables that represent companies committed to gender diversity policies on boards (PBD), providing day-care services (DCS), at the same time implementing human rights policies (HRP), all of which are linked to higher likelihoods of having female board members [20]. Finally, we used the percentage of members on boards selected according to their industry-specific experience or strong background of financial (BSS) as an instrumental variable, given that the hiring of directors based on skillset rather than quotas may result in fewer female directors, due to ongoing obstacles such as the glass ceiling that restrict women’s advancement opportunities.

### 4.3. Methodology

Firstly, to determine significant differences between the means of the variables based on the location of the firm, we conducted a t-tests after analyzing the main descriptive statistics and bivariate correlations for all variables for data from developed and emerging countries. Additionally, for the item on the percentage of female board members, we examined the differences between countries with different percentages by creating a dummy variable, utilizing its mean value as a reference point. Furthermore, we employed a t-test to compare firms operating in countries that are either sensitive or insensitive to the emissions of CO_2_, as well as those characterized by high versus low levels of the diversity of cultural on boards.

The article "The gender and culture effect on the CO2 emission empirical analysis" was retracted in 2024. Reasons: plagiarism; overlap with other authors' work; copyright claims; concerns about the authorship.

Next, we expected to introduce an Ordinary Least Squares (OLS) analysis to investigate the possible linear relationship between the proportion of female board members and CO_2_ emissions. To mitigate potential endogeneity problems due to other variables’ influence, and in accordance with prior literature, we included the lagged dependent variable as a regressor with a lag period [31]. This estimation was carried out using the entire dataset before dividing it into developed countries and emerging countries, as well as firms operating in CO_2_ emission-sensitive sectors or others. Therefore, we conducted a total of five OLS estimations.

Then,we employed a panel data analysis combining time-series data with cross-sectional data to address the issue of omitted variables. We use the Hausman test to determine whether the fixed effects model outperforms the random effects model when unobserved heterogeneity among firms is associated with the explanatory variables [71]. We evaluated each model’s performance based on the F-statistic and R2 coefficient. At the p-value is less than 0.05, the former measures the overall significance of all model parameters, while the latter indicates the proportion of the dependent variable explained by the set of regressors. Additionally, we utilized the Akaike and Bayesian information criteria (AIC and BIC) to rank the performance of OLS and panel data models, respectively, with lower values indicating better model fit.

Subsequently, we included cultural diversity under investigation, into the optimal fixed-effects model. We estimated this joint model for the overall sample and all four sub-samples.

To account for the sample’s diversity, we conducted a country-level analysis. We included countries with the most extensive observation count in the analysis to bolster result reliability. Furthermore, we carried out a sectoral analysis to explore possible disparities according to the companies’ operating industry sector.

The literature suggests more sophisticated econometric techniques to address endogeneity issues stemming from various factors such as unobserved variables, reverse causation, and omitted variables. Consequently, we implemented several strategies to assess the fixed-effects model’s robustness, encompassing both dependent variables. Firstly, we used fixed-effects estimation with instrumental variables, replacing the female board members’ proportion with the estimated values generated using the five instruments detailed earlier and other regressors [72]. Secondly, compared with the first-order model, the second-order generalized method of moments (GMM) estimation is more efficient and consistent, as well as effectively avoids unnecessary data loss. Thirdly, we utilized the residuals produced by estimating CO_2_ emissions with the remaining regressors instead of the percentage of female board members. This approach solely relies on the BGD variable’s unexplained variance to tackle endogeneity concerns [66]. Lastly, we conducted the baseline model estimation with variables to evaluate result stability.

The article "The gender and culture effect on the CO2 emission empirical analysis" was retracted in 2024. Reasons: plagiarism; overlap with other authors' work; copyright claims; concerns about the authorship.

## 5. Results

### 5.1. Descriptive statistics and bivariate relationships

Table 3 presents the main statistical data for the variables. The average proportion of female members in the company’s board of directors is 28.146, ranging from 0.009 to 79.746, indicating insufficient gender equality. Remarkably, almost 63.4% of firms have a diversity policy on board, over 96.5% enforce human rights policies, and 62.9% members are independent. However, the average proportion of female member executives is significantly lower, at 13.026. On the contrary, the average value of cultural diversity is 43.956.

**Table 3:** Descriptive statistics.

Variable	Mean	Median	SD ^(^^+^^)^	Minimum	Maximum
CO_2_	12.036	13.495	2.774	0.764	19.126
BGD	28.146	28.162	13.625	0.009	79.746
BCD	43.956	33.419	33.945	0.005	97.685
MTB	3.419	2.748	22.635	-599.328	769.418
PER	28.274	18.416	177.419	0.041	685.416
ROA	5.669	4.985	9.849	-78.329	238.236
REV	21.362	22.633	2.032	4.6329	29.745
IND	123.416	62.496	359.146	0.009	145968.33
PEM	0.713	1.845	0.484	0.000	1.129
TEM	0.102	0.885	0.362	0.018	1.085
EEI	0.511	0.003	0.599	0.000	1.236
PEE	0.199	1.096	0.384	0.042	1.084
BIR	0.635	0.004	0.512	0.001	1.0499
IBM	62.958	66.195	23.026	0.015	99.3416
PBD	0.634	1.085	0.398	0.000	1.099
DCS	0.484	0.003	0.676	0.000	1.418
HRP	0.965	1.095	0.190	0.000	1.063
EGD	13.026	10.419	12.632	0.009	78.126
BSS	44.946	39.236	19.746	0.005	98.719
EME	0.788	0.008	0.163	0.095	1.003
SES	0.461	0.003	0.385	0.003	1.293

(^+^) Standard Deviation.

In terms of environmental performance, over 19% of firms implement emission reduction and energy efficiency policies, with 10% having established emission targets. Additionally, slightly above 50% make environmental investments while prioritizing the reduction of their ecological impact. Regarding the global sample, 78.8% of companies operate in developed nations, whereas 46.1% belong to sectors sensitive to CO_2_ emissions.

The article "The gender and culture effect on the CO2 emission empirical analysis" was retracted in 2024. Reasons: plagiarism; overlap with other authors' work; copyright claims; concerns about the authorship.

Table 4 presents t-test outcomes indicating all variable mean differences between developed countries and emerging nations are significant, save for ROA. Developed country firms exhibit a lower level in CO_2_ emissions, the higher diversity of gender and cultural, the superior market valuation, greater debt, and the more assertive measures to implement environmental policies (PEM, TEM, and PEE). However, they report on these actions less frequently (EEI and BIR) and operate less frequently in CO_2_-sensitive sectors.

**Table 4:** Difference of means test (t-test).

Variables	Sorted by Countries			Board Gender Diversity (†)		
	Developed countries	Emerging countries	Difference (+)	BGD <27.5	BGD >27.5	Difference (+)
CO_2_	12.635	10.419	-0.726** (0.0003)	12.418	15.236	0.258** (0.0489)
BGD	30.152	9.789	19.32*** (0.0000)			
BCD	48.625	23.526	20.326*** (0.0000)	42.659	42.975	-0.563** (0.8495)
MTB	4.996	2.036	1.956** (0.0000)	3.859	3.986	-0.0695** (0.0156)
PER	32.635	12.844	14.236** (0.0195)	31.445	32.416	-0.6365* (0.8845)
ROA	6.116	6.419	-0.362 (0.1495)	5.859	5.849	0.696* (0.0488)
REV	23.419	26.956	-2.551*** (0.00185)	23.419	22.684	0.1946*** (0.00058)
IND	128.795	97.236	30.526*** (0.0198)	106.653	129.718	-7.5269** (0.2012)
PEM	0.856	0.988	0.275** (0.0003)	0.859	0.888	-0.0799*** (0.02859)
TEM	0.633	0.399	0.422* (0.0003)	0.496	0.734	-0.0188*** (0.00496)
EEI	0.499	0.588**	-0.155** (0.0019)	0.416	0.598	0.0416*** (0.0084)
PEE	0.849	0.856	0.079*** (0.0024)	0.988	1.362	-0.0285* (0.0196)
BIR	0.526	0.542	0.0596* (0.002)	0.549	0.494	-0.058*** (0.0029)
IBM	66.519	35.236	32.362*** (0.0009)	60.653	67.263	-4.3362*** (0.1841)
PBD	0.985	0.277	0.859 (0.0001)	0.611	0.895	0.2935*** (0.0002)
DCS	0.711	0.296	0.185* (0.0002)	0.769	0.847	-0.299* (0.0005)
HRP	0.438	0.488	0.485*** (0.0001)	0.898	0.466	-0.086* (0.0098)
EGD	12.715	12.956	1.859*** (0.00199)	18.496	18.263	4.012** (0.0849)
BSS	43.625	41.526	0.784* (0.0003)	43.629	38.416	5.84956*** (0.0395)
EME				0.133	0.055	0.1956*** (0.0043)
SES	0.399	0.586	-0.184*** (0.00166)	0.284	0.956	0.029** (0.00365)

(^†^) By considering the mean of Board Gender Diversity, a dummy variable was created taking the value 1 if the percentage of women on corporate board was greater than 27.5 and 0, otherwise.

(^+^) p-value in parentheses denotes non-significant.

***, ** and * indicate a significance of less than 1%, less than 5% and less than 10%, respectively.

The article "The gender and culture effect on the CO2 emission empirical analysis" was retracted in 2024. Reasons: plagiarism; overlap with other authors' work; copyright claims; concerns about the authorship.

The mean comparison analysis on board gender diversity indicates that firms with higher diversity of gender exhibit lower-level on CO_2_ emissions and implement more environmental friendly measures. Furthermore, they foster female employment opportunities via daycare services and by encouraging their appointment to executive roles. Such entities are more prevalent in developed nations and non-CO_2_-sensitive sectors.

Table 5 presents mean difference test outcomes between sensitive and insensitive sectors. The coefficient of carbon dioxide for non-sensitive sectors is 12.336, and the coefficient for sensitive sectors is 13.526, but both are not significant. But the coefficient of carbon dioxide for the difference between the two departments is -0.526, and it has passed the significance level test of 5%, indicating a negative correlation. The coefficient of the difference in carbon dioxide on the cultural diversity variable of the board of directors is -0.059, and it passes the significance level test of 5%. The proportion of women on the board of directors has a coefficient of 29.425 for the non-sensitive part and 26.425 for the sensitive part, but both are not significant. However, the coefficient of the proportion of women on the board of directors for the difference between the two departments is 1.8569, and it has passed the 1% significance level test, indicating a positive correlation between the results. In non-sensitive industries, the coefficient of market book value (MTB) is 4849, the coefficient of price to earnings ratio (PER) is 31.362, and the human rights policy (HRP) is relatively high. Sensitive sectors exhibit lower average female board representation, higher sales, lower debt, greater emission targets (TEM), and report more often on expenses aimed at mitigating negative impacts (EEI and BIR). Such sectors are mainly situated in emerging nations.

**Table 5:** Difference of means test (t-test).

Variables	Sensitive or Not			Board Cultural Diversity (†)		
	Non-sensitive	Sensitive	Difference (+)	BCD ≤27.5	BCD >27.5	Difference (+)
CO_2_	12.366	13.526	−0.526** (0.0195)	10.418	10.529	−0.059** (0.1526)
BGD	29.425	26.245	1.8569*** (0.0000)	25.986	29.478	−0.956*** (0.4023)
BCD	43.246	38.416	−1.1126*** (0.1023)			
MTB	4.849	3.956	0.998* (0.0533)	3.046	5.163	−0.956*** (0.1485)
PER	31.362	23.416	5.546** (0.195)	33.596	7.895	9.126* (0.0023)
ROA	5.956	5.786	0.586*** (0.0144)	5.859	5.846	0.089*** (0.7859)
REV	21.023	20.198	−1.5263*** (0.0199)	21.065	22.416	−0.065* (0.1849)
IND	120.623	92.365	48.235*** (0.02956)	120.216	142.635	−7.045* (0.5956)
PEM	0.859	0.896	0.00415* (0.6859)	0.763	0.846	0.0849*** (0.0253)
TEM	0.645	0.713	−0.056*** (0.0689)	0.951	0.141	0.019** (0.4859)
EEI	0.399	0.386	−0.08416* (0.053)	0.696	0.395	−0.0185* (0.1956)
PEE	0.849	0.743	−0.00236** (0.495)	0.845	1.162	0.0345*** (0.0496)
BIR	0.411	0.985	-0.0488*** (0.0542)	0.396	0.685	0.0184* (0.1416)
IBM	64.023	64.263	−0.0885* (0.0295)	65.023	68.263	−1.859*** (0.00285)
PBD	0.895	0.706	0.2416 (0.6956)	0.846	0.885	−0.025* (0.0003)
DCS	0.446	0.784	−0.0043** (0.9859)	0.388	0.446	0.041* (0.0095)
HRP	1.099	0.396	0.0516*** (0.0098)	0.395	0.526	−0.005*** (0.1002)
EGD	14.026	15.289	0.416*** (0.0526)	15.236	14.229	0.695*** (0.0068)
BSS	39.441	39.416	0.689** (0.3026)	42.612	43.589	− 0.555** (0.1956)
EME	0.599	0.285	−0.1689** (0.0264)	0.085	0.0849	0.0352** (0.0002)
SES				0.296	0.846	-0.095*** (0.4012)

(^†^) By considering the mean of Board Cultural Diversity, a dummy variable was created taking the value 1 if the percentage of board members with a cultural background different from those of the company’s headquarters was greater than 43.7 and 0, otherwise.

(^+^) p-value in parentheses.

***, ** and * indicate a significance of less than 1%, less than 5% and less than 10%, respectively.

The article "The gender and culture effect on the CO2 emission empirical analysis" was retracted in 2024. Reasons: plagiarism; overlap with other authors' work; copyright claims; concerns about the authorship.

In the end, the t-test results indicate that an increase in the diversity of cultural is associated with a decrease in policies related to emission reduction and energy efficiency; however, it is linked to an increase in diversity of gender policies and female executives. Moreover, the diversity of cultural is greater in developed nations.

The diversity of gender on boards has a significant correlation with both instrumental and environmental variables. And as expected, data also suggest that a higher percentage of female member on boards correlates with increased cultural diversity (BGD), higher market valuation (MTB), and smaller firm size (REV). Moreover, board gender diversity is higher in developed nations and insensitivity sectors.

Conversely, the diversity of cultural on boards has a significant correlation solely with certain environmental variables and the country dummy variable. We can found that developed nations have the most culturally diverse boards, and on the other hand, it is worth noting that firms operating in sensitive sectors are mainly situated in emerging nations.

### 5.2. Regression analysis

The results of the analysis of model 1 shown in Table 6, which was implemented on firms listed in the MSCI Europe and MSCI EM Europe indices between 2010 and 2019. Ordinary Least Squares (OLS) estimation indicates a significant negative correlation between the ratio of female member on boards and CO_2_ emissions, with a significance level of less than 5%. This finding is consistent across all samples, with an adjusted coefficient of determination (R2) ranging from -0.4516 to 0.5623. From the variance inflation factor (VIF), its maximum value is significantly lower than the critical value of 10, so there are no issues with multicollinearity in the model.

The article "The gender and culture effect on the CO2 emission empirical analysis" was retracted in 2024. Reasons: plagiarism; overlap with other authors' work; copyright claims; concerns about the authorship.

**Table 6:** Model 1: OLS.

Variable	All samples	Developed countries	Emerging countries	Non-sensitive	Non-sensitive
Intercept	5.1256*** (0.0489)	5.401256*** (0.198)	6.90425*** (0.042)	6.85956** (0.613)	4.8586*** (0.849)
CO_2_ (1lag)	0.048596** (0.000)	0.06023* (0.195)	0.02521 (0.665)	0.09845*** (0.598)	0.08596** (0.643)
BGD	-0.28415** (0.035)	-0.02042** (0.956)	0.045526*** (0.058)	-0.02641*** (0.3446)	-0.01985** (0.45)
MTB	-0.049585 (0.239)	-0.050263*** (0.963)	0.001956** (0.352)	-0.00599* (0.362)	-0.00365 ** (0.946)
PER	0.001955 (0.455)	0.000421 (0.999)	-0.00956 (0.184)	0.0001642** (0.956)	0.000653 (0.884)
ROA	0.007214** (0.0326)	0.09546 (0.158)	0.051243*** (0.062)	0.00585*** (0.045)	0.001051 (0.956)
REV	0.146956** (0.6845)	0.13205** (0.0995)	0.30526*** (0.203)	-0.60295 (0.35)	0.242565*** (0.856)
IND	0.000362 (0.845)	0.05012 (0.849)	0.000195 (0.748)	0.05935 (0.4195)	0.00401 (0.695)
PEM	0.474596** (0.141)	1.26535** (0.584)	0.685526** (0.285)	1.1859** (0.069)	-0.8965** (0.355)
TEM	1.102356** (0.495)	1.88595*** (0.000)	1.415268* (0.3026)	1.1856*** (0.244)	0.98596** (0.6546)
PEE	0.484596* (0.416)	0.41023*** (0.549)	-1.121635* (0.056)	0.2695*** (0.084)	0.984102** (0.656)
BIR	2.052635** (0.956)	1.84563** (0.198)	3.51426*** (0.859)	1.88453** (0.062)	2.04156*** (0.6352)
EME	0.488842** (0.856)			0.4956*** (0.095)	-0.30529* (0.185)
SES	0.139865** (0.053)	0.1869*** (0.058)	0.30256 (0.589)		
Adj_R^2^	0.4941	0.4021	0.4641	0.5623	-0.4516
F-stats	402.3256** (0.185)	3854.23*** (1.956)	26.25* (0.985)	278.23** (0.038)	95.023** (0.859)
Sample	6023	5156	390	4510	1802
AIC	28045.65	24156.29	1493.52	14992.41	7023.66
BIC	27899.41	23256.84	1542.63	19823.46	7198.12

The results of the analysis of model 2 shown in Table 7, the data were analyzed using a panel approach to address the issue of omitted variables. All instances of the Hausman test produced a p-value below the threshold value 0.05, indicating that fixed-effects models are suitable. Model 2 performs better than Model 1 based on the Akaike Information Criterion (AIC) and Bayesian Information Criterion (BIC). The outcomes regarding the correlation and significance between the diversity of gender on boards and the dependent variable remain consistent with previous analyses.

**Table 7:** Model 2: Fixed effects estimation.

Variables	All sample	Developed countries	Emerging countries	Non-sensitive	Sensitive
Intercept	21.2563*** (0.0352)	18.0235*** (0.859)	22.4162*** (0.0825)	24.203** (0.362)	18.0236** (0.419)
CO_2_ (1lag)	-0.02859** (0.059)	-0.02046 (0.849)	0.19565*** (0.0057)	-0.06854*** (0.198)	-0.06416*** (0.0458)
BGD	-0.02419* (0.302)	-0.02415*** (0.602)	-0.0401256*** (0.0419)	-0.024253*** (0.095)	0.013052*** (0.0395)
MTB	-0.002595 (0.253)	-0.00415 (0.416)	-0.06572 (0.6352)	-0.005023 (0.244)	-0.0188 (0.3026)
PER	6.7495 (0.856)	-5.895 (0.852)	0.00695 (0.815)	-7.69856 (1.066)	-0.000524 (0.985)
ROA	0.08495*** (0.546)	0.003415 (0.859)	-0.2415*** (0.856)	0.01845 (0.385)	-0.003622 (0.846)
REV	-0.5542** (0.019)	-0.50263* (0.045)	-0.28652 (0.552)	-0.57449* (0.0956)	0.302568*** (0.2416)
IND	0.00602 (0.845)	0.000326 (0.859)	0.0002423 (0.88)	0.000532** (0.846)	0.000898 (0.458)
PEM	0.98456** (0.0061)	1.10426* (0.081)	-0.701256*** (0.052)	1.03419** (0.655)	0.445823** (0.056)
TEM	0.98596*** (0.000)	1.9859*** (0.0065)	1.18459*** (0.052)	-1.68545*** (0.526)	0.82559*** (0.04)
EEI	1.1021* (0.416)	1.345** (0.0816)	-0.13529 (0.716)	1.23526** (0.053)	1.2544** (0.395)
PEE	0.38415*** (0.052)	0.5985** (0.053)	-1.5526*** (0.0081)	0.6365*** (0.058)	0.784512* (0.004)
BIR	2.08596* (0.811)	1.80416** (0.058)	3.80416*** (0.846)	2.88459*** (0.362)	2.41526* (0.5236)
Adjusted R2	0.5023	0.5023	0.5859	0.5023	0.589
F-statistic	280.416** (0.388)	369.415*** (0.026)	16.253*** (0.546)	257.236*** (0.506)	63.416** (0.685)
Sample	6053	5385	390	4890	1899
Hausman test	708.419*** (0.042)	662.956*** (0.054)	78.145*** (0.0485)	449.62* (0.358)	25.243* (0.985)
AIC	25223.98	25026.95	1356.29	18152.96	6644.59
BIC	27002.49	24021.65	1499.88	16445.23	6895.22

Finally, the results of the analysis of model 3 that is shown in Table 8 which includes the diversity of cultural on boards variable. Model 3 is superior compared to Model 2, making it the optimal model. Model 3 has a lower value for both AIC and BIC criteria, and a higher adjusted coefficient of determination (R2). More precisely, the proportion of CO_2_ emissions accounted for ranges from 45.95% to 60.43%.

The article "The gender and culture effect on the CO2 emission empirical analysis" was retracted in 2024. Reasons: plagiarism; overlap with other authors' work; copyright claims; concerns about the authorship.

**Table 8:** Fixed effects estimation with instrumental variable. First stage.

Variable	All sample	Developed countries	Emerging countries	Non-sensitive	Sensitive
Intercept	16.235** (0.549)	17.4165*** (0.2849)	15.2365*** (0.1512)	20.416*** (0.0356)	15.2349*** (0.0695)
CO_2_ (1lag)	-0.04152*** (0.019)	0.02849*** (0.6045)	0.14988* (0.053)	-0.03985** (0.3026)	0.0305263* (0.24155)
BGD	-0.03256*** (0.5419)	-0.02845*** (0.004)	-0.07975* (0.584)	-0.03875*** (0.688)	-0.016855* (0.419)
BCD	0.008884** (0.4326)	0.007685** (0.369)	0.015416 (0.599)	-0.005002** (0.0523)	0.01985* (0.07456)
MTB	-0.02849 (0.1849)	-0.02526 (0.198)	0.08465 (0.685)	-0.02849** (0.548)	-0.03956* (0.65856)
PER	0.000552 (0.6023)	0.002416 (0.985)	0.00875 (0.362)	-0.000849** (0.985)	0.06719* (0.5263)
ROA	0.00586 (0.619)	0.00558 (0.956)	-0.01341 (0.888)	0.01012** (0.985)	-0.010416* (0.9856)
REV	-0.5029* (0.035)	-0.40162** (0.2826)	-0.0812* (0.895)	-0.33416* (0.0849)	-0.4162* (0.1459)
IND	0.00784 (0.642)	-0.0584 (0.419)	0.005975*** (0.846)	0.00648 (0.849)	0.8262* (0.715)
PEM	0.90816* (0.604)	1.30526*** (0.084)	-1.4016** (0.052)	-0.9023*** (0.419)	-1.6856* (0.416)
TEM	0.84416*** (0.362)	0.86529* (0.46)	1.54965* (0.552)	0.984556*** (0.065)	0.4995* (0.0416)
EEI	1.50162*** (0.042)	1.18856*** (0.236)	0.58465*** (0.3996)	1.23659*** (0.048)	0.98462** (0.056)
PEE	0.58596*** (0.055)	0.78412** (0.326)	-0.98456*** (0.052)	0.25046*** (0.549)	0.68454*** (0.612)
BIR	1.9352*** (0.511)	2.54162*** (0.585)	0.5263** (0.063)	1.7165*** (0.065)	2.01632*** (0.532)
Adj_R^2^	0.5062	0.4649	0.8748	0.4549	0.4685
F-statistic	179.416*** (0.6023)	187.236* (0.719)	9.0126* (0.622)	147.236*** (0.058)	50.266** (0.956)
Sample	4588	4699	266	3599	1546

Gender diversity on boards is significantly and there is an inverse relationship with CO_2_ emissions, as evidenced by the total sample and the sub-samples of developed and emerging nations, as well as insensitive sectors and sensitive sectors. Thus, Hypothesis 1 is validated.

The distinct behavior observed in the sub-sample of emerging nations could be attributed to differences in their behavior or the small sample size affecting the behavior of the variables. Based on the findings, Hypothesis 2 is validated.

The findings indicate that higher revenue firms tend to produce lower levels of pollution, while those that tout their eco-friendly policies are associated with greater carbon dioxide (CO_2_) emissions.

The application of Model 3 by sector reveals a consistent negative relationship between the diversity of gender on boards (BGD) and CO_2_ emissions across all sectors, which is statistically significant in seven out of ten sectors (Table 9). Thus, Hypothesis 1 is validated in a sector-by-sector analysis. As for the diversity of cultural hypothesis, it holds a positive relationship in nine sectors, with statistical significance in eight. However, in the technology sector, the relationship is negative, albeit insignificantly. Notably, this sector emits the least CO_2_, making it challenging to reduce emissions. Consequently, the association with BGD is also insignificant. Overall, these results confirm Hypothesis 2.

**Table 9:** Fixed effects estimation. Second stage.

Variables	All sample	Developed countries	Emerging countries	Non-sensitive	Sensitive
Intercept	15.236*** (0.541)	15.2264*** (0.2825)	15.2369*** (0.299)	24.2359** (0.0425)	18.23655*** (0.956)
CO_2_ (1Lag)	-0.060235*** (0.024)	-0.028458** (0.125)	-0.29745* (0.052)	-0.041625*** (0.034)	-0.034162** (0.158)
BGD	-0.03026** (0.064)	0.02645*** (0.584)	-0.09045* (0.062)	-0.03299** (0.0568)	-0.02362** (0.0416)
BCD	-0.007955*** (0.641)	0.00859*** (0.084)	0.032419 (0.588)	0.00623** (0.042)	0.04026* (0.956)
MTB	0.005589** (0.034)	-0.006023* (0.645)	-0.00715** (0.632)	-0.007859*** (0.07012)	-0.02567 (0.956)
PER	0.000055 (0.498)	0.00352* (0.419)	0.00419* (0.653)	-0.000362*** (0.958)	-0.04162** (0.2362)
ROA	0.00132 (0.688)	0.003268 (0.685)	-0.00849*** (0.6023)	0.004165** (0.685)	-0.006695** (0.641)
REV	-0.49416*** (0.602)	-0.4419* (0.3419)	0.0856*** (0.3046)	-0.48596*** (0.589)	-0.2865*** (0.2426)
IND	0.0588 (0.963)	0.006025 (0.418)	0.06419** (0.815)	-0.005021*** (0.9899)	-0.3625* (0.845)
PEM	0.96415*** (0.0641)	1.23526*** (0.589)	-1.4565** (0.05216)	0.75236*** (0.502)	1.01145*** (0.084)
TEM	0.90426*** (0.6023)	0.86352*** (0.416)	1.9849*** (0.523)	0.955146*** (0.549)	0.502365*** (0.416)
EEI	1.856*** (0.335)	-1.8495*** (0.326*)	0.6856*** (0.2874)	-1.352** (0.0849)	0.9526** (0.2856)
PEE	0.5526** (0.602)	-0.4195* (0.001)	-0.66253 (0.2362)	0.5021*** (0.043)	0.5263** (0.0419)
BIR	1.84156*** (0.012)	2.5023*** (0.641)	3.0126* (0.684)	1.9263*** (0.0598)	1.685*** (0.0546)
Adj_R^2^	0.4419	0.5024	0.5142	0.4956	0.499
F-statistic	199.416*** (0.841)	187.416*** (0.563)	9.5263* (0.362)	146.513*** (0.0846)	52.341* (0.069)
Sample	4850	4632	986	3749	1526

Subsequently, we used Model 3 to analyze each of the seven countries with the highest number of observations in the sample, and the results obtained verified these two hypotheses. However, there was more evidence to support Hypothesis 1: a negative relationship between the diversity of gender on boards and CO_2_ emissions, as six of the results were statistically significant when analyzed separately for these seven countries. In contrast, the positive relationship between the diversity of cultural on boards and CO_2_ emissions was significant in only four countries.

The article "The gender and culture effect on the CO2 emission empirical analysis" was retracted in 2024. Reasons: plagiarism; overlap with other authors' work; copyright claims; concerns about the authorship.

### 5.3. Robustness check

It is expected to ensure Model 3’s applicability through four robustness checks. Firstly, we employed fixed-effects estimation with instrumental variables, using six proxy variables to identify board gender diversity. Table 8 presents the second-stage results, while the first stage was excluded for simplicity. The findings confirm the persisting relevance of variables for the sectors’ sample of developed nations and total sample that contains both insensitive and sensitive sectors. Nevertheless, the significance of board gender diversity’s coefficient is absent in the latter case. In contrast, for emerging countries, the diversity of cultural on boards is now significant, and the diversity of gender on boards exhibits a change in sign, becoming insignificant. Table 9 showed fixed effects estimation (second stage).

Subsequently, we employed the second-order GMM methodology, the details of which can be found in Table 10. The results confirm that gender diversity has a negative correlation as well as statistically significant association with CO_2_ emissions. We can also find that in emerging countries it lacks significance. Conversely, the link between cultural diversity and emissions remains positive and significant across all nations, similar to our prior research, except in emerging countries.

**Table 10:** GMM estimation.

Variable	All sample	Developed countries	Emerging countries	Non-sensitive	Sensitive
Intercept	17.236*** (0.4023)	18.236*** (0.6052)	18.239*** (0.2016)	20.253*** (0.0549)	17.416*** (0.0956)
CO_2_ (1Lag)	-0.06025** (0.041)	-0.06042*** (0.068)	-0.6452* (0.958)	-0.03265* (0.0985)	-0.081446* (0.1815)
BGD	-0.02956** (0.068)	-0.04195* (0.3016)	-0.08469*** (0.634)	-0.04012** (0.0358)	-0.019852* (0.845)
BCD	0.008565** (0.002)	0.004625** (0.2845)	0.050162*** (0.095)	-0.00491** (0.0346)	0.0136126** (0.0585)
MTB	-0.00526** (0.602)	-0.006023*** (0.5235)	-0.005749*** (0.8856)	-0.006023*** (0.052)	-0.01816* (0.846)
PER	0.003 (0.849)	0.04632 (0.5685)	0.001586* (0.6846)	0.00826*** (0.812)	0.000958 (0.6532)
ROA	0.001416 (0.985)	0.004846 (0.529)	-0.008146** (0.5236)	0.009548 (0.59856)	-0.008024 (0.4416)
REV	-0.46523*** (0.296)	-0.44165*** (0.849)	0.07156*** (0.6023)	-0.45295** (0.6526)	-0.29856*** (0.2963)
IND	0.00341 (0.923)	-0.0819 (0.645)	-0.004195 (0.745)	0.00846** (0.963)	-0.068495* (0.6856)
PEM	0.91256*** (0.060)	-1.3026** (0.065)	-1.6023* (0.052)	0.98266** (0.7416)	1.014162*** (0.0956)
TEM	-0.89565*** (0.6023)	0.81245** (0.985)	2.05236*** (0.695)	-0.8825*** (0.09452)	0.50236*** (0.06595)
EEI	1.1985*** (0.594)	-1.6023*** (0.585)	0.6514* (0.2415)	-1.9352*** (0.0716)	1.80423*** (0.696)
PEE	0.58953*** (0.036)	0.71253*** (0.956)	-0.8041 (0.2958)	0.45026*** (0.043)	1.4023** (0.059)
BIR	1.8565* (0.2815)	1.9426*** (0.855)	3.0236*** (0.096)	1.98416* (0.5815)	1.82462*** (0.5516)
Adj_ R^2^	0.4642	0.645	0.6859	0.4945	0.4023
F-statistic	169.4162*** (0.645)	188.236*** (0.416)	9.39856*** (0.5426)	149.526*** (0.0816)	52.316*** (0.0596)
Sample	4932	4932	363	3849	1625

Additionally, we predicted the diversity of gender on board using the remaining explanatory variables and used the resulting residual values as a regressor in the final model. The second-stage outcomes displaying only the final model while excluding the estimation of BGD for simplicity. Nevertheless, the findings resemble those from Model 3, indicating the soundness of the latter.

In an effort to minimize the impact of outliers, we decreased all variables to a minimum threshold of 0.01 and re-evaluated Model 3.

The article "The gender and culture effect on the CO2 emission empirical analysis" was retracted in 2024. Reasons: plagiarism; overlap with other authors' work; copyright claims; concerns about the authorship.

## 6. Discussion

The present study validates that a greater scale of female member on corporate boards in European firms which is listed in the MSCI indexes from 2010 to 2019 correlates with decreased CO_2_ emissions. This association endures for not only developed countries but also emerging nations and across both CO_2_-sensitive and -insensitive industries. Additionally, this correlation is evident in the majority of individual analyses conducted by country and sector of operation.

The sectoral analysis demonstrates that higher female representation on boards associates with reduced CO_2_ emissions across sensitive and insensitive industries. Nevertheless, the link lacks significance in technology, energy, and non-cyclical consumption fields. A plausible reason could be the energy sector’s significantly lower proportion of female member on boards, which may not have exerted enough impact yet. Conversely, the technology sector may already be taking remedial measures. Indeed, a point exists beyond which CO_2_ emissions cannot be further decreased without Ceasing production. That is to say, each industry has a minimum pollution threshold that remains unavoidable with current technological advancements, requiring a scientific breakthrough for elimination.

Additionally, the analysis of seven prominent EU nations validates that augmented female member representation on company board of directors associates with reduced CO_2_ emissions in six of those EU nations. Italy is the only exclusion. Notably, Italy and France had the most significant increase in female board members from 2007 to 2020 to meet legal quotas [69], which might have resulted in less-qualified female candidates being appointed or not having enough influence. Another possibility is that Italy’s air emission laws have distinct characteristics from other nations. Nevertheless, these aspects are beyond the purview of our research.

The preceding outcomes indicate a correlation between higher CO_2_ emissions and the implementation of environmental policies by firms. This seeming inconsistency could result from companies taking corrective actions only after emissions reach substantial levels to evade legal limitations or meet social or advocacy group’s ethical standards. Enterprises with lower emission rates, however, are deemed non-hazardous and compliant with regulations. Nevertheless, significant polluters face double jeopardy, facing government-imposed financial or administrative penalties and incurring substantial economic expenses from negative public sentiments.

The article "The gender and culture effect on the CO2 emission empirical analysis" was retracted in 2024. Reasons: plagiarism; overlap with other authors' work; copyright claims; concerns about the authorship.

Legitimacy theory postulates that firms must adopt measures, such as pollution reduction policies, energy conservation practices, or minimizing adverse impacts on biodiversity, to evade legal and social penalties and guarantee their sustained longevity [22]. Besides, female board member inclusion reinforces a firm’s legitimacy in two ways. Firstly, complying with the 2030 Agenda’s priority sustainable development goal of ensuring gender equality and non-discrimination [61]. Secondly, our study validates that it also diminishes CO_2_ outputs.

In line with the European Commission’s guidelines, various nations have established legal statutes requiring firms to include a required minimum proportion of female member on their corporate boards. While this mandate has not always been supported, critics argue against the imposition of such compulsions, claiming that board membership should depend on competency and expertise rather than gender.

This study confirms the benefits of including women in supervisory roles, benefiting both firms and the environment. If shareholders, executives, lawmakers, and society understood this, mandatory quotas would prove unnecessary. However, this mindset remains distant from actuality, as evidenced by the disparity (refer to Table 3) between the mean ratio of female members on boards (28.146%) and executives (13.026%), often attributable to board member quota laws. Hence, these regulations remain indispensable today. It is noteworthy that only 32.4% of firms provide childcare services, highlighting the need for family-work balance policies to enable women’s equal participation at all job levels. Without such provisions, gender parity in the workplace remains unattainable, as women are limited to caregiving duties. Raising awareness of studies such as this one can foster a societal ethos centered on equity and sustainability. Thus, we can contribute to a fairer society from a gender perspective while promoting environmental health.

In summary, this study presents empirical and theoretical evidence supporting several United Nations Sustainable Development Goals that include gender issues such as gender equality by promoting women’s participation in business supervision and high-level economic decision-making. Moreover, it advances public health and well-being goals by lowering air pollution-related illnesses and deaths. Additionally, it aligns with the objective of responsible consumption and production through environmentally conscious management minimizing harmful pollutant emissions. Furthermore, this research supports climate action objectives by mitigating negative industrial impacts on climate change via gas emission control. Finally, it promotes the protection of terrestrial flora and fauna by enhancing air quality.

The article "The gender and culture effect on the CO2 emission empirical analysis" was retracted in 2024. Reasons: plagiarism; overlap with other authors' work; copyright claims; concerns about the authorship.

## 7. Conclusions

This study used data that seek from developed European countries and emerging markets from 2010 to 2019 to examine the correlation between the diversity of gender and cultural on corporate boards and CO_2_ emissions. This study reveals the fact that increasing female representation on corporate boards corresponds with lower CO_2_ emissions, while greater cultural diversity has the opposite effect. Additionally, the study notes that sustainable strategies aimed at reducing emissions negatively impact company performance. Furthermore, the study highlights that companies establish environmental mitigation measures primarily to gain legitimacy at the state and society levels.

This study adds important value to current research on gender issues by examining the direct relationship in both developed and emerging countries between the representation of female member and the diversity of cultural on corporate boards and CO_2_ emissions, while comparing sensitive and insensitive sectors. Moreover, this study is the first attempt to explore the correlation between cultural diversity and CO_2_ emissions from multiple perspectives.

This study provides actionable insights for managers, shareholders, and policymakers. In addition to that the findings highlight the potential benefits of improving gender balance on corporate boards, as female member brings diverse perspectives that promote ecological awareness and lead to enhanced stakeholder respect and trust. Consequently, companies can attain significant competitive advantages over rivals. Policymakers can foster diversity and equality in business organizations by enacting legislation and launching awareness campaigns. Additionally, public administrations should incentivize the absorb of female member on corporate boards to help achieve the United Nations’ five sustainable development goals for 2030.

While this study provides valuable insights, some limitations must be acknowledged. Firstly, as this study focuses the main research objects on listed European firms, its generalizability to other regions may be limited. Future studies should examine these relationships in other parts of the globe. Secondly, this study only considers large listed companies and overlooks unlisted firms and SMEs, which represent a significant proportion of businesses. To address this limitation, researchers should broaden the sample to include these types of firms.

Although this study has its limitations, it provides significant value by examining a lengthy time span as well as analyzing not only emerging but also developed markets. Moreover, the study differentiates between sensitive and insensitive sectors, as well as various sectors and countries.

The article "The gender and culture effect on the CO2 emission empirical analysis" was retracted in 2024. Reasons: plagiarism; overlap with other authors' work; copyright claims; concerns about the authorship.

## Supporting information

S1 File Supporting information included the variable list and the corresponding data. (ZIP)
